# A Comparative Study on the Clinical Efficacy of Stereotaxic Catheter Drainage and Conservative Treatment for Small and Medium Amount Intracerebral Hemorrhage in the Basal Ganglia

**DOI:** 10.1155/2022/7393061

**Published:** 2022-09-27

**Authors:** Junhui Yuan, Yansong Lv, Shaowei Zhang, Yongpeng Li, Xi Jiao

**Affiliations:** Department of Neurosurgery, Sanmenxia Central Hospital, Sanmenxia, Henan 472000, China

## Abstract

The incidence rate and fatal disability rate of cerebral hemorrhage increase year by year. At present, most patients with a hematoma volume of ≤20 mL are treated conservatively by internal medicine. With the development of the stereotactic technique, it has been widely used for the treatment of cerebral hemorrhage in clinics. This study compared the clinical differences between stereotactic surgery and conservative treatment for small- and medium-sized cerebral hemorrhages. The results show that stereotactic hematoma evacuation is more effective than conservative treatment in the treatment of medium and small intracerebral hemorrhages in the basal ganglia. It can accelerate the resolution of hematoma and improve the neurological function and quality of life of patients, which is worthy of clinical promotion and application.

## 1. Introduction

Spontaneous intracerebral hemorrhage (SICH) refers to intracerebral hemorrhage caused by spontaneous rupture of large and small arteries, veins, and capillaries of the brain due to various reasons under nontraumatic factors [1, 2]. Hypertension is the most common predisposing factor for SICH, and the risk of SICH disease in hypertensive patients increases with age [3]. SICH with a hematoma volume of less than 30 mL is considered to be a moderate-to-small-volume SICH. In the past, it was considered that surgery was not required for small and medium-sized SICH, and conservative medical treatment was the first treatment option for patients [4]. However, more and more data showed that although patients with small- and medium-sized SICH had low blood loss and low mortality, the neurological function of the patients will be significantly damaged, and the recovery of neurological function of patients with conservative medical treatment is poor [5, 6]. Therefore, some scholars have suggested that for small- and medium-sized SICH diseases, auxiliary surgical schemes can be adopted, such as small bone window craniotomy, craniotomy, and endoscopic surgery.

Brain stereotactic technology has been put forward for more than 100 years. It has experienced a long period from experiment to instrument setting to clinical application, and its development tends to be mature. Stereotaxic technology includes frame positioning technology, frameless brain stereotaxic technology, cube orientation technology, and neuronavigation technology. Previous studies have shown that the injury caused by open surgery might offset the efficacy of hematoma removal to varying degrees, but hematoma removal based on stereotaxic techniques may be more helpful in improving the prognosis [7, 8]. Recently, stereotaxic technology has been used in the treatment of SICH, known as stereotactic catheter drainage [9, 10]. In the present study, 146 patients with small and medium-sized cerebral hemorrhages in the basal ganglia were selected, which was designed to compare the clinical effects of stereotactic catheter drainage and conservative drug therapy in patients with small and medium amounts of intracerebral hemorrhage in the basal ganglia.

## 2. Methods and Materials

### 2.1. Patients and Grouping

A total of 146 patients with small- and medium-sized cerebral hemorrhages in the basal ganglia who were admitted to our study from January 2019 to December 2021 were included. According to different treatment protocols, the patients were divided into 2 groups, control group and research group (73 patients in each group). There was no statistically significant difference in the general data between the two groups, and they were comparable (*P* > 0.05). All studies in the present study were approved by the hospital ethics committee, and patients and their families voluntarily signed the hospital-related informed consent.

### 2.2. Inclusion Criteria

(1) Age ≥18 years old; (2) small and medium amount intracerebral hemorrhage in the basal ganglia by head CT; (3) no previous history of SICH; (4) no anticoagulants were taken 2 weeks before joining the group; (5) patients with hypertension history; (6) and patients admitted to hospital within 24 hours after symptoms appeared.

### 2.3. Exclusion Criteria

(1) Patients with other surgical contraindications such as coagulation disorders; (2) combined with other serious diseases, such as malignant tumor, liver, kidney, or other organ dysfunctions; (3) history of mental illness, intellectual disability, or communication impairment; (4) history of taking anticoagulants or immunosuppressants; (5) history of traumatic brain injury, cerebrovascular malformation, cerebral aneurysm, and stroke; (6) alcohol addiction or drug addiction; and (7) coexisting systemic diseases, such as autoimmune diseases, chronic infectious diseases, or uremia.

### 2.4. Treatment Protocol

Patients in the control group received conservative drug treatment, including symptomatic treatment such as oxygen inhalation, blood pressure stabilization, dehydration, and prevention of bedridden-related complications.

Patients in the research group received stereotaxic surgery. In brief, patients were placed in a supine position before the operation and given local anesthesia after disinfection of the surgical site. The headframe was installed, and then a CT examination of the head was performed. The center of the hematoma or the surgical target was determined on the computer, and the *X*, *Y*, and *Z* values were calculated. After the location of the surgical incision is determined, the dura is drilled and incised. An intraoperative stereotactic navigation device was installed, and the drainage tube was placed according to the procedure. During the operation, 5–15 mL of clot was slowly aspirated. After surgery, 30,000 units (5 mL) of urokinase were injected into the hematoma cavity to provide adequate drainage of the hematoma. Finally, a reexamination of the head CT is performed and the drainage tube is removed within 1 to 3 days after surgery.

### 2.5. Baseline Data Collection

Collect the clinical data of patients through the hospital electronic medical record system, including gender, age, course of hypertension, hematoma volume, GCS score of admission, location of hematoma, comorbidities, and degree of paralysis of the limb.

### 2.6. Hematoma Volume Measurement

At admission and 1, 3, 7, 14, and 30 days after treatment, all patients underwent head CT examination, and the largest high-density area of the CT section was selected to measure the longest and widest diameters of the hematoma. Brain hematoma calculation formula: hematoma volume (mL) = 1/2 × longest diameter (cm) × widest diameter (cm) × CT slice thickness (cm) *x* number of CT slices [11].

### 2.7. Observation Indicators

1. Clinical prognosis. Length of hospital stay, number of complication cases, diseased limb muscle strength on 30th day after treatment (level 4–5 on the Lovett scale), and the Glasgow outcome scale (GOS) on 90th day after treatment [12].
2. Neurological assessment. We used the National Institute of Health Stroke Scale (NIHSS) [13] and the modified ranking rating scale (mRS) [14] to evaluate the neural function of patients before treatment and at 7, 14, 30, and 90 days after treatment. Among them, the NHISS score ranged from 0 to 42, and the higher the score, the more serious the nerve defect was. The maximum score of mRS was 6 points, and 0 points meant no symptoms at all. A score of 1 indicates that, despite the symptoms, the insured has no obvious disability and is able to complete all the frequently engaged work and activities. 2 points mean slightly disabled, unable to complete all work and activities, but able to handle personal affairs without the help of others. 3 points indicate moderate disability and the need for help from others, but no help when walking. 4 points represent severe disability, inability to walk without the help of others, and inability to take care of oneself. A 5 indicates severe disability, bedridden, incontinence, need for continuous care, and a need to be looked after more than 24 hours a day. 6 points mean dead.
3. Daily life recovery. Before treatment and at 7, 14, 30, and 90 days after treatment, we used the Modified Barthel Index (MBI) to evaluate the patient's functions of daily living and activities [15]. The highest score of the MBI scoring criteria was 100 points, with 61–99 points indicating mild need dependence, 41–60 points indicating moderate dependence, and ≤40 points indicating severe dependence.

### 2.8. Statistical Analysis

Data in the present study were analyzed by SPSS 20.0 software (SPSS Inc., Chicago, USA). The measurement data were expressed as ($\bar{x}$ ± S) and the *t*-test was performed. The count data were expressed as percentage (%) using the *χ*^2^ test, and *P* < 0.05 indicated that the difference was statistically significant.

## 3. Results

### 3.1. Baseline Data

The baseline data including gender, age, course of hypertension, hematoma volume, GCS score of admission, location of hematoma, comorbidities, and degree of paralysis of the limb between the two groups were comparable with no significant difference (Table 1).

### 3.2. Clinical Outcome

During 90-dayfollow-up, there were no deaths in two groups. At the same time, the time of hematoma vanish, the number of complication cases and the time of hospital stay in the research group were significantly lower than those in the control group (*P* < 0.05), while the number of cases where the degree of paralysis of the limb on the diseased side recovered to level 5 on the 30th day and the number of GOS scores >5 on the 90th day in the research group were all significantly higher than those in the control group (*P* < 0.05) (Table 2).

### 3.3. Hematoma Volume

Patients in two groups were followed up with head CT at 1, 3, 7, 14, and 30 days after treatment to calculate the hematoma volume by the Tada formula. As shown, the hematoma of the patients in the research group began to drain 3 days after treatment, while that in the control group was 30 days after treatment. In conclusion, the hematoma volume in the control group was significantly higher than that in the research group on days 1, 3, 7, 14, and 30 after treatment (*P* < 0.05) (Table 3).

### 3.4. Neurological Score

Patients in two groups were followed up on neural function using the NIHSS scale and the mRS scale before treatment and at 7, 14, 30, and 90 days after treatment. As shown, there was no significant difference in the NIHSS score and the mRS score before treatment between the control group and the research group (*P* < 0.05), while the scores of NIHSS and mRS in the research group at 7, 14, 30, and 90 days after treatment were all significantly lower than those in the control group (*P* < 0.05) (Table 4).

### 3.5. Daily Life Recovery

Patients in two groups were followed up on activities of daily living and activities using the MBI scale before treatment and at 7, 14, 30, and 90 days after treatment. As shown, there was no significant difference in MBI scores before treatment between the control group and the research group (*P* > 0.05), while MBI scores in the research group at 7, 14, 30, and 90 days after treatment were all significantly higher than those in the control group (*P* < 0.05) (Table 5).

## 4. Discussion

Intracerebral hemorrhage has the characteristics of “high morbidity, high recurrence rate, high disability rate, and high fatality rate.” The basal ganglia area is a relay station for nerve fiber conduction and is also the spontaneous brain. At present, it is considered that a hematoma volume of >30 ml is the indication for craniotomy, while for patients with a hematoma volume of ≤30 ml, conservative drug therapy is generally used [16]. However, previous studies have shown that patients with 15–30 mL of cerebral hemorrhage in the basal ganglia region may develop hemiplegia and aphasia [17]. Because the hematoma cannot be removed in time during the conservative treatment, the brain tissue and nerve fiber bundle will be compressed for a long time, leading to irreversible changes in the nerve fiber bundle [18]. At the same time, the existence of compression will also cause cell ischemia and hypoxia, secondary pathological changes and necrosis, and toxic effects on the surrounding cells. In addition, the decomposition of blood produces hemosiderin, which aggravates the edema of surrounding tissues and aggravates the compression, further aggravating the fiber bundle injury [19]. Therefore, after conservative treatment, it is difficult for such patients to restore their motor and language functions to the expected effects, which will impose a great burden on the family economy and life in the future. The persistent existence of hematoma is the starting factor of this series of vicious circles. Only when the etiology disappears will the vicious circle be broken and the prognosis of patients will be improved.

Through clinical practice, it is generally believed that the advantages of stereotactic hematoma evacuation are as follows: ① it is simple to operate and quick to operate. ② The localization is accurate, and the application range is wide. The inserted drainage tube can accurately reach any target set before surgery. ③ The patients with hypertensive intracerebral hemorrhage are mostly middle-aged and elderly people, and most of them are complicated with heart, lung, diabetes, and other diseases, which will seriously affect the life and quality of life of the patients after the operation [20]. However, this technique can be operated under local anesthesia. The preparation time and operation time are short, with no obvious contraindication. The trauma is small. Hematoma drainage is thorough when urokinase is used to dissolve hematoma. The patient has a short bed rest time, rapid recovery, and few complications. Additional brain injury caused by surgical striking and repeated traction caused by the traditional craniotomy operation can be avoided. ④ After successful stereotactic catheterization, 60% of the hematoma was suctioned out, and the disease would be relieved. In line with the diagnosis of hypertensive intracerebral hemorrhage, the hematoma should be quickly and effectively removed to reduce secondary brain injury, which is conducive to the rescue of early patients with cerebral hernia [21]. ⑤ A single catheter placement can be used for multiple drug injections, irrigation, and drainage, and the position and depth of the catheter placement can be adjusted according to the extraction of hematoma. Repeated puncture and catheterization are avoided, and the probability of intracranial infection and rebleeding is reduced. This study found that in the research group treated with stereotactic surgery, the average disappearance time of hematoma, the number of complications, and hospital stay were significantly lower than those in the control group. The number of cases in which the degree of limb paralysis on the affected side recovered to Grade 5 on the 30th day and the GOS score >5 on the 90th day were significantly higher than those in the control group, and the edema degree and mass effect around the hematoma in patients were also significantly lower than those in patients treated with medication. This indicates that stereotactic surgery can improve the patient's disorder of consciousness, reduce the related complications, start rehabilitation treatment earlier, and increase the GOS score of the patient in 90 days.

In addition, we also found that the recovery of neurological function and daily activity after surgery in the research group receiving stereotactic therapy was significantly better than that in the control group receiving conservative treatment, which was consistent with the research results by Huang et al. [22]. This further confirmed that the postoperative neurological recovery of small- and medium-sized SICH patients treated by stereotactic surgery was significantly superior to conservative treatment. The reason is that stereotactic surgery is conducive to the rapid removal of hematoma, which can reduce the mass effect, alleviate the compression on brain tissue, and reduce the damage to neurons, the pyramidal tract, and glial cells around hematoma caused by various toxic substances released during the solidification, liquefaction, and decomposition of hematoma, thereby reducing the incidence of secondary damage to brain tissue.

However, through clinical practice, we have found some noteworthy places. The operation timing of applying stereotactic techniques to cerebral hemorrhage is controversial. Because the internal hemorrhage is not stable for 6 h after the onset of cerebral hemorrhage, the operation at this time will increase the risk of rebleeding. Therefore, it is not recommended to conduct stereotactic operations during this period.

## 5. Conclusion

Stereotactic hematoma evacuation is more effective than conservative treatment in the treatment of medium and small intracerebral hemorrhages in the basal ganglia. It can accelerate the resolution of hematoma and improve the neurological function and quality of life of patients, which is worthy of clinical promotion and application. However, this study is only a cohort study, the measurement indicators are highly subjective, and it fails to provide a causal conclusion. It also does not conduct in-depth research on clinical communication skills, but it provides more ideas for in-depth research on stereotactic hematoma evacuation in the future.

## Figures and Tables

**Table 1:** Baseline data of two groups.

Baseline data	Control group (*n* = 73)	Research group (*n* = 73)	*t*/*χ*^2^	*P*
Gender (*n*)				
Male	43	46	0.259	0.611
Female	30	27		
Age (years)	63.58 ± 9.38	65.24 ± 8.13	0.628	0.327
Course of hypertension (years)	7.03 ± 2.15	7.08 ± 2.08	1.124	0.105
Hematoma volume (mL)	18.91 ± 4.02	18.19 ± 3.34	0.956	0.297

GCS score of admission				
3–12	53	52	0.034	0.854
13–15	20	21		

Location of hematoma				
Thalamus	23	21	0.559	0.906
Outside the putamen	30	33		
Inner side of putamen	12	13		
Caudate nucleus	8	6		

Comorbidities (*n*)				
No	31	27	0.535	0.765
Diabetes	9	11		
Coronary heart disease	33	35		

Upper extremity muscle strength (*n*)				
Level 1	18	15	0.353	0.838
Level 2	20	21		
Level 3	35	37		

Lower extremity muscle strength (*n*)				
Level 1	15	12	0.536	0.755
Level 2	21	20		
Level 3	37	41		

*Note.* GCS, Glasgow Coma Scale.

**Table 2:** Comparison of observation indicators related to clinical outcomes between the two groups.

Observation indicators	Control group (*n* = 73)	Research group (*n* = 73)	*t*/*χ*^2^	*P*
Hematoma vanish (days)	24.62 ± 4.35	3.36 ± 1.57	29.328	<0.001
Complication occur (*n*)	20	9	5.207	0.023
Hospital stay (days)	23.31 ± 3.81	17.34 ± 4.95	13.567	<0.001
Diseased limb muscle strength at 30th day (level 4–5) (*n*)	29	47	8.892	0.003
GOS score >5 at 90th day (*n*)	45	60	7.631	0.006

*Note. GOS, Glasgow Outcome Scale.*

**Table 3:** Comparison of hematoma volume at different times between the two groups ($\bar{x}$ ± *s*, mL).

Time	Control group (*n* = 73)	Research group (*n* = 73)	*t*/*χ*^2^	*P*
1st day	19.65 ± 4.14	15.65 ± 3.05	5.138	0.031
3rd day	19.61 ± 4.06	5.36 ± 2.24	18.637	<0.001
7th day	19.08 ± 3.94	2.15 ± 0.69	23.157	<0.001
14th day	13.38 ± 2.15	0.00 ± 0.00	34.392	<0.001
30th day	2.95 ± 1.01	0.00 ± 0.00	10.927	<0.001

**Table 4:** Comparison of NIHSS score and mRS score at different times between the two groups ($\bar{x}$ ± *s*, score).

Observation indicators	Control group (*n* = 73)	Research group (*n* = 73)	*t*	*P*
NIHSS score				
Before treatment	9.33 ± 2.82	9.51 ± 2.35	0.698	0.301
7th day	9.08 ± 2.35	8.04 ± 2.19	4.269	0.042
14th day	7.56 ± 2.03	6.67 ± 1.82	5.638	0.021
30th day	6.87 ± 1.96	4.98 ± 1.68	10.957	<0.001
90th day	4.82 ± 1.35	3.56 ± 1.12	6.351	0.013

mRS score				
Before treatment	4.85 ± 0.92	4.90 ± 0.89	0.719	0.264
7th day	4.18 ± 0.82	3.81 ± 0.76	4.038	0.047
14th day	4.01 ± 0.86	3.14 ± 0.62	4.537	0.038
30th day	3.06 ± 0.79	1.91 ± 0.65	6.956	0.008
90th day	2.84 ± 0.97	1.25 ± 0.54	7.329	<0.001

*Note.* NIHSS, National Institute of Health Stroke Scale. mRS, Modified Ranking Rating Scale.

**Table 5:** Comparison of MBI score at different times between the two groups ($\bar{x}$ ± *s*, score).

Time	Control group (*n* = 73)	Research group (*n* = 73)	*t*	*P*
7th day	22.53 ± 9.56	21.86 ± 8.93	0.834	0.297
14th day	29.61 ± 13.32	38.21 ± 10.34	7.935	<0.001
30th day	47.86 ± 13.25	75.62 ± 16.82	13.628	<0.001
90th day	60.45 ± 14.57	85.67 ± 11.53	19.147	<0.001

*Note.* MBI, Modified Barthel Index.

## Data Availability

The data used and/or analyzed during the current study are available from the corresponding author.
